# Seasonal Changes in Pesticide Residues in Water and Sediments from River Tano, Ghana

**DOI:** 10.1155/2022/8997449

**Published:** 2022-04-30

**Authors:** Jackson Adiyiah Nyantakyi, Samuel Wiafe, Osei Akoto

**Affiliations:** ^1^Environmental Protection Agency, P.O. Box GS 166, Goaso, Ahafo Region, Ghana; ^2^Sunyani Technical University, Sunyani, Ghana; ^3^Kwame Nkrumah University of Science and Technology, Kumasi, Ghana

## Abstract

Pollution due to pesticide residues has been reported in the downstream of the Tano Basin in the rainy season and has been attributed to the anthropogenic activities upstream. However, data on the seasonal variations in pesticide residues in the upstream of Tano Basin are limited. Seasonal variations in 13 organochlorine pesticide residues, 8 organophosphorus pesticide residues, and 5 synthetic pesticide residues in water and sediment samples of River Tano upstream were assessed through extraction and Varian CP-3800 gas chromatography equipped with a CombiPAL Auto sampler set at ionization mode electron impact methods. Significantly higher pesticide residues were detected in water and sediment samples in the rainy season than the dry season. Permethrin (rainy: 0.007 ± 0.01 mg/kg; dry: 0.008 ± 0.02 mg/kg) and profenofos (rainy: 0.021 ± 0.02 mg/kg; dry: 0.026 ± 0.01 mg/kg) showed higher dry season concentrations in the sediment samples. Two isomers of lindane (*δ*-HCH = 0.059 ± 0.24 *μ*g/L; *γ*-HCH = 0.002 ± 0.01 *μ*g/L) were detected in the water in the rainy season, but 3 were detected in the sediment samples (*δ*-HCH = 0.004 ± 0.12 mg/kg; *γ*-HCH = 0.003 ± 0.01 mg/kg; aldrin = 0.001 ± 0.01 mg/kg) suggesting possible illegal use. The detected pesticide residual levels in both water and sediment samples were lower than the maximum residual levels in water and sediment. The Chemical Control and Management Centre of the Environmental Protection Agency should check possible faking and adulteration of banned organochlorine pesticides.

## 1. Introduction

Increasing pesticide use and misapplications of pesticides along river basins pose serious threats to aquatic ecosystems [1, 2]. Increasing incidence of vector diseases is contributing to increasing use of pesticides [3–5]. Pesticides are mostly used by farmers in the rainy season to control pests [6–8]. Most buffer zones which have been created along river banks to protect them from runoffs have been compromised through anthropogenic activities [9]. It has been established that only 5% of the applied pesticides reach the targets and the remaining 95% settle on nontarget organisms and water bodies [10, 11]. Pesticides in surface water are known to pose serious environmental and public health-related problems [11–16]. Thus, human exposure to pesticides through ingestion of contaminated water are known to cause health-related problems such as birth defects, endocrine disruption, nerve related problems, and mutation [3, 17, 18].

Diverse types of pesticides are used worldwide, but the most widely used in developing countries are insecticides [1]. Organophosphorus, organochlorine pesticides, and synthetic pyrethroids are usually used for pest control [19, 20]. However, organochlorine pesticides have been banned in Ghana and in some Western countries due to their toxicity, bioaccumulation, extensive half-life, low polarity, high stability, and persistence in the environment [3, 17]. In spite of the ban on the use of OCP by the Stockholm convention, they are illegally used in some developing countries making the ban ineffective [21]. For example, about 4.99 × 10^6^ tons of OCPs are produced and distributed annually for agricultural purpose in China [22, 23]. In the year 2014, China alone consumed about 1.8 million tons of pesticide, Argentina consumed about 200 thousand tons of pesticides, USA consumed 125,000 tons, India consumed 110,000 tons, and Mexico consumed 98,000 tons [24].

Ghana imported about 13,000 metric tons of pesticides in 2006 and 13,000 metric tons in 2019 for agricultural and health issues [25]. The use of these pesticides is misused or misapplied due to low supervision and sensitization by extension officers [1]. The most commonly applied pesticides in Ghana are synthetic pyrethroids (SPPs) and organophosphorus (OPs) [17, 18]. Studies conducted in some basins in Ghana have shown some appreciable levels in residues of pesticide in water, sediment, and fish [26, 27].

River Tano plays unique and complex ecological roles that influence the structures and functions of their catchment areas in Ghana and La Côte d'ivoire [28]. It serves as a drinking water source for over 2.4 million people living in the basin catchment [28, 29]. However, the downstream water quality of the river is currently being threatened by pesticide pollution driven by increased farming activities in the rainy season and degraded buffer zone upstream [9]. Pesticide contamination in the upstream of the Tano River has been suspected over the years because of the compromised buffer zone due to farming activities, but data on this are limited [29]. The river receives high suspended solids through runoff which may serve as conduits for pollutants including pesticide residues in the river [28, 30]. Data on the pesticide residues in the upstream of the Tano Basin are needed for water quality supervisors and strategy producers to make an informed decision, but this information is limited. The aim of this study was to assess pesticide residues in the upstream of River Tano resulting from variation in seasons. The study provides valuable information on pesticide residue concentrations in the upstream of the Basin.

## 2. Materials and Methods

### 2.1. Study Area

The study covers the source of the Tano River at Tuobodom in the Bono East Region, to the downstream of Ashanti Region. Eight districts/municipalities are found in the study area. They include Techiman North district, Techiman municipality, Sunyani municipality, Tano North municipality, Asutifi North district, Asutifi South district, Asunafo North municipality, and Asunafo South district. The predominant anthropogenic activities within the study area include agriculture, commercial, industrialization, and human settlement which have compromised the buffer zone created to protect the basin [9, 30]. The vegetation is damp green and semideciduous biological precincts [31]. Dry and rainy seasons are experienced in the study area. The raining season happens between April and October, whereas the dry season happens between November and March every year [9]. The normal yearly precipitation is in the range of 1,140–1,300 mm for each year, and temperature is in the range of 25.8^o^C [32]. The general stickiness ranges between 75 and 85% consistently. The yearly evapotranspiration is around 1,500 mm with the yearly spillovers being 2,774 m^3^ [28, 31].

### 2.2. Study Design

Thirty-six sediment and water samples each at nine sites in the Tano River were periodically collected between November and March 2016 (dry season) and April and October 2017 (rainy season). The river from the source to the point where it enters Ashanti was sectioned into nine sampling zones (S_1_, S_2_, S_3_, S_4_, S_5_, S_6_, S_7_, S_8_, and S_9_). A sampling point was sited at the downstream of a given anthropogenic activity that leads to the release of pesticides into the river (Figure 1 and Table 1). Garmin 62SC Geographical Positioning System (GPS) was employed to coordinate and map out the sampled points (Figure 1).

13 organochlorines pesticide (OCP) residues, 8 organophosphorus pesticide (OP) residues, and 5 synthetic pyrethroids pesticide residues (SPP) were studied. The OCPs included *γ*-HCH, *δ*-HCH, *α*-HCH, heptachlor, aldrin, chlordane, *β*-HCH, *α*-endosulfan, *β*-endosulfan, dieldrin, endrin, p,p-DDT, and p,p-DDE. The OPs were methamidophos, diazinon, fenitrothion, malathion, chlorpyrifos, pirimiphos-methyl, profenofos, and parathion. The SPPs were allethrin, permethrin, deltamethrin, cyfluthrin, and fenvalerate.

### 2.3. Sampling and Sample Treatment

Brand new plastic bottles were used to collect the water samples. Collection of water samples followed the methodology previously described by Chapman [33]. One litre of water was sampled at each sampling location and stored in the sample bottle (the bottle was rinsed with water from the river before taking the samples).

All the samples in their respective bottles were branded and preserved in a cooler laden with ice as previously described by Nyantakyi [29]. At each of the selection locations, replica samples were collected and well kept.

With the aid of the Van Veen Grab Sampler, sediment samples were collected by dropping it into the river sediments (that is from the river bank and then at about 1.20 m into the river). The two grab samples were mixed, and 200 g of the sediment was collected as previously described by Bhuyan et al. [34]. The sediment samples were placed in a brand new polyethene zip lock bag which had previously been cleaned with sanitized water and rinsed with the river water as prescribed by Gereslassie et al. [35]. The polyethene zip lock bag containing the sample was labelled and preserved in a cooler with ice as previously prescribed by Okoya et al. [36]. The procedure was repeated for the remaining sample locations. Duplicate samples were collected at all the sampling sites [29]. The residue of pesticides in water and sediment samples was carried out in the laboratory of Ghana Standards Authority, Accra, Ghana.

### 2.4. Extraction and Clean-Up of Pesticides in Water

Liquid-liquid extraction (LLE) method previously described by Afful et al. [37] and Nyantakyi [29] was used in this study. 50 mL of sampled water was poured into a separating funnel, and 50 mL mixture of hexane and acetone in the ratio of 2 : 1 was added and shaken vigorously for 10 min. The mixture was made to settle, and the organic layer was drained into another container. Another 50 mL of hexane-acetone mixture was added to the sample and shaken for another 20 min. The new organic layer was added to the previous organic layer. A rotary evaporator was used to concentrate the extract to 2 mL. A clean column packed with 4 g of silica and of Na_2_SO_4_ was then set up and conditioned with 10 mL of hexane. 4 mL hexane was used to elute the packed extract on the column. The eluted sample was then concentrated to near dryness and taken up in 2 mL ethyl acetate and transferred with a Pasteur pipette into GC vials for pesticide analyses.

### 2.5. Extraction and Clean-Up of Pesticides in Sediment Samples

The extraction and clean-up of pesticides in sediment samples followed the methodology previously described by Akoto et al. [38]. Sediment samples were dried overnight after which 10 g of the sample was poured in a conical flask and 60 mL of solvent (hexane-acetone in 2 : 1 ratio) and sonicated for 20 min. The supernatant was filtered, and 60 mL of hexane-acetone combination was added to the sample and resonicated for another 20 min. The supernatant was then filtered and added to the previous one and then concentrated on a rotary evaporator to about 20 mL. A column was then cleaned, set up, packed with 4 g of silica and 2 g of Na_2_SO_4_, and conditioned with 10 mL of hexane. Using a Pasteur pipette, the concentrated filtrate was then loaded on to the column and eluted with 5 mL of hexane. The eluted sample was concentrated to near dryness and was taken up in 2 mL of ethyl acetate and kept in GC vial ready for analysis.

### 2.6. Analysis of Extracts for Pesticide Residues

Analyses of extracts for pesticide residues in water and sediment samples followed the method previously described by Akoto et al. [38] and Graíño et al. [39] at Ghana Standards Authority (GSA) pesticide residue laboratory in Accra, Ghana. Varian CP-3800 gas chromatography equipped with a CombiPAL autosampler set at ionization mode electron impact (EI) was used for the pesticide residues. The chromatographic conditions were set as follows: a ZB-5MS (30 m × 0.25 mm × 0.25 *μ*m) column from Phenomenex (Torrance, CA, USA) was utilized. The injector temperature was 300°C. The injection was splitless, and the injection volume was 1.0 *μ*L. The transfer line and source temperature were set at 300°C. Nitrogen gas was used as the carrier gas at a flow of 1.0 mL per min. The oven temperature was initially at 40°C for 2 mins and then increased at the rate of 9°C/min until 300°C for 3 minutes. The identification of the pesticide residues was premised on the comparison of relative time of retention and acknowledged standards and further quantified by the peak area of the external standard method.

### 2.7. Quality Control (QC) and Quality Assurance (QA)

Strict QC and QA protocols were observed in terms of precision, accuracy, representativeness, and completeness in order to ensure that the results produced were scientifically acceptable. All instruments used in this study were calibrated and validated using specificity method as previously described by El-Gawad [40]. Deionized organic-free water samples were used as blanks. In addition, precision of the extraction procedures was evaluated by carrying out recovery analysis of the liquid-liquid extraction (LLE) which was expressed as relative standard deviation (RSD %) as previously described by LCP (1996). Recovery experiments were used to assess the accuracy and precision by spiking the samples with pesticides at 0.01 and 0.05 mg/L for the water samples and 0.01 and 0.05 mg/kg for the sediment samples at *n* = 5 interval as previously described by Pindado et al. [41]. Intermediate precision was also assessed by analysing 5 fortified samples at 0.1 mg/L and 0.1 mg/kg respectfully for water and sediment samples, respectively. The results were expressed as percentages.

### 2.8. Data Analysis

R software was used in analysing the data [29]. The standard deviation and means for the respective classes of pesticide residue (OCPs, SPPs, and OPs) were computed for each sampling site. A *t*-test was used to compare the means between the two seasons of pesticide levels in water and sediment [42]. The priority was to establish the significant relationship in group means between levels of pesticides between both seasons for the water and sediment. In this analysis, *p* value < 0.05 was taken to be statistically significant [43]. Again, principal component analysis (PCA) was carried out employing JMP statistical software v. 10 (SAS Institute) to determine the distribution pattern of pesticides in water. Eigenvalue >1 by varimax rotation served as extracts for the principal components.

## 3. Results and Discussion

### 3.1. Precision and Accuracy

The results for the precision and accuracy are shown in Table 2 The European Commission [44] suggests in their guidelines (SANCO/12571/2013) that RSD (%) ≤20 considered suitable and acceptable values for multiresidue methods. In this assessment, the RSD values were all <20%. This indicates that the results are reliable and acceptable. The pesticide recovery percentages for the pesticides ranged from 98% to 104% in the accuracy and precision assessment (Table 2). This suggests that the pesticide recovery in the water and sediment samples are considered satisfactory [44].

### 3.2. Seasonal Variation in OPs Residues in Sediment and Water Samples

Table 3 shows the variations in the season of OP in sediments and water. The results showed that the levels of OPs residues in water and sediment samples for the rainy season were generally above the dry season samples. In the water samples, parathion pesticide residues in the rainy season (0.268 ± 0.01 *μ*g/L) were significantly above dry season (0.027 ± 0.02 *μ*g/L) samples (*p* < 0.05). In the sediment samples, parathion, methamidophos, and pirimiphos-methyl residues in the rainy season were significantly higher than the dry season. This may be due to higher runoffs with increased precipitation of suspended solids containing the pesticide residues in the runoff. In the Songhua River and Afram River in Ghana, Wang et al. [11] and Senyo et al. [27], respectively, reported on higher parathion residues in the rainy season. This was similar to the observed parathion residues in the rainy season in this study. In the Achelous River in Greece, Stamatis et al. [45] reported on significantly higher OP residue levels in summer (dry season) than winter (rainy season) which were in contradiction to the observations made in this study. Generally, the major source of OP pesticide residues to surface water bodies is agricultural runoffs and drift from application of OPs through spraying [46]. Increased OP pesticide applications in the rainy season as well as activities of farming may result in higher OP levels in the rainy season.

Comparison between OP levels in water and sediment samples revealed that OP residues in water were generally higher than the sediment samples to suggest that OP pesticides are hydrophilic and vastly soluble in water [47, 48].

### 3.3. Variations in Season of Pyrethroid Residues

The results for the seasonal variations in synthetic pyrethroids pesticide (SPP) residues in water and sediment samples are shown in Table 4. The results showed that the levels of SPP in both water and sediment samples were generally low. This may be due to the fact that SPP residues breakdown when they are exposed to sunlight [17]. The results further showed that the levels of allethrin, permethrin, deltamethrin, and cyfluthrin pesticide residues in the wet season were significantly above the corresponding levels in the dry season for the water samples. The highest SPP residues recorded in the rainy season was permethrin (0.019 ± 0.02 *μ*g/L), while the least residue level was fenvalerate (0.007 ± 0.01 *μ*g/L). In the dry season, the highest SPPs residue was recorded by allethrin (0.012 ± 0.01 *μ*g/L), and the least dry season concentration was 0.001 ± 0.00 *μ*g/L by fenvalerate. In the sediment samples, the levels of SPPs residues in the rainy season were insignificantly higher than the corresponding dry season levels (Table 3). Again, the SPP residue in sediment samples were lower than the levels in water to suggest the hydrophilic nature of SP [13, 49]. The presence of SPP residues in water and sediment samples may be attributed to higher farming activities along the course. Senyo et al. [27] reported on SPP residues ranging between 0.01 and 2.135 *μ*g/L in River Afram in Ghana which was higher than the observed concentrations in this study. The levels of SPP residues which were similar to the observed residue levels were also reported by Riaz et al. [50] in River Chenab in Pakistan. Higher levels of SPPs residues in the rainy season may suggest that SPP use was higher in the rainy season where farming activities were high with increased agricultural runoffs [49].

### 3.4. Variations in Season in Organochlorine in Sediment and Water Samples

Table 5 shows the variations in season in OCPs residue in sediment and water sample. In the water samples, two isomers of lindane *δ*-HCH (0.059 ± 0.24 *μ*g/L) and *γ*-HCH (0.002 ± 0.01 *μ*g/L) were recorded in the rainy season, but the levels were lower than the limits of detection <0.01 *μ*g/L in the dry season. In the sediment samples, three OCP residues were detected in the rainy season. They were aldrin (0.001 ± 0.01 mg/kg), *δ*-HCH (0.004 ± 0.12 mg/kg), and *γ*-HCH (0.003 ± 0.01 mg/kg). The rest of the OCP studied were not found sediment and water samples. In the Saruria River in Bangladesh, Hasanuzzaman et al. [51] also reported that chlordane, *α*-endosulfan, *β*-endosulfan, dieldrin, endrin, p,p-DDT, and p,p-DDE were not detected. This was similar to what was observed in this study. Again, the levels of *δ*-HCH in water were relatively higher than the corresponding levels in the sediment samples to suggest it is very soluble in water. The level of *γ*-HCH in the sediment samples were above the water samples to suggest its hydrophobic properties [52].

The residues of pesticides found in the water samples were both hexachlorocyclohexane (HCH). The half-life of HCH and its isomers range from 20 days to 15 months (FAO [53]. This may suggest that the isomers of HCH which were detected in this study were recently applied. The use may be put into malaria control, agricultural, or industrial [3]. Generally, if the ratio of *δ*-HCH to *γ*-HCH concentrations in sediment is below 3, it suggests that the source of HCH to the aquatic ecosystem is a new input [29, 54]. In this study, the ratio of *δ*-HCH to *γ*-HCH was 1.3 which suggests that the HCH source to River Tano is a fresh input. However, Akoto et al. [17] reported on a ban on OCP use in Ghana since 1986 and freshly applied OCPs are not expected in water and sediment samples. However, Lugushie [55] reported aldrin, chlordane, and heptachlor in the midstream of (Asutifi South district) of River Tano. Nguyen et al. [56] reported on some levels of heptachlor, aldrin, dieldrin, and endrin found in sediment and water samples of Don Nai River in Vietnam. Senyo et al. [27] detected 14 OCPs in the Afram Basin. Fianko et al. [57] detected 8 OCPs in River Densu. Akan et al. [58] detected appreciable levels of OCP residues in River Benue in Nigeria. These may suggest illegal use of OCPs. Due to its high potency and efficacy, OCPs are adulterated resulting in multiple active ingredients in the adulterated OCPs in the market and the environment with the consequent environmental and public health effects [59]. In the downstream of the Tano Basin Lugushie [55] reported on appreciable levels of 20 OCP residues in the Tano Basin. However, contrary to his study, only 3 of the OCP residues were detected.

### 3.5. Principal Composite Analysis for Organophosphorus Pesticide Residues

The results of the principal composite analysis (PCA) for organophosphorus residues of pesticide in the Tano Basin are in Table 6 and Figure 2. The results showed that 2 components with eigen factors greater than 1 were extracted. The first component accounted for 60% of the loading and was dominated by all OPs circled as “a.” They were profenofos, malathion, diazinon, chlorpyrifos, and pirimiphos-methyl. The second component was dominated by OPs circled in “b” which included parathion, fenitrothion, and methamidophos. The OPs with the same association possibly will suggest they are coming from the same source or have similar properties [60]. The probable source may include industrial, agricultural, and municipal runoffs [35].

## 4. Conclusion

The study assessed the seasonal variations of thirteen organochlorine pesticides, eight organophosphorus pesticide residues, and five synthetic pesticide residues in 36 each of sediment and water samples from Tano River. All the pesticides studied were detected in the water and sediment samples except organochlorines pesticides residues, where only 2 were detected in water samples and 3 in the sediment samples in the rainy season. The rainy season concentrations of the pesticide residues were above the dry season mean concentrations except for permethrin and profenofos that recorded higher levels in the dry season. Higher concentrations in the rainy season were attributed to higher farming activities with increased volumes of runoffs from the agricultural activities along the river banks. The levels of pesticides residues detected in the water samples were above the corresponding levels in the sediment samples for both seasons. The levels of all the pesticide residues for both dry and rainy seasons were within the maximum permissible pesticide residual levels in water. Principal composite analysis revealed strong association among profenofos, malathion, diazinon, chlorpyrifos and pirimiphos-methyl which suggested similarity in properties. A second component dominated by parathion, fenitrothion, and methamidophos was extracted to suggest a possible source to the Tano River which may possibly be due to agricultural activities There should be strict enforcement of the buffer zone policy to ameliorate further deterioration of the Tano River pesticide residue water quality. Current use of banned pesticides including the organochlorines was suspected. In view of their persistence in the environment coupled with their high toxicity, the Chemical Control and Management Centre of the Environmental Protection Agency should improve on the monitoring of pesticide use, faking, and adulteration of banned pesticides in Ghana.

## Figures and Tables

**Figure 1:** Map of Ghana showing the upstream of the Tano Basin, sampling sites, and land use.

**Figure 2:** Principal composite analysis of OP residues in water samples from River Tano.

**Table 1:** GPS locations of the sampling sites and distances between them.

Sampling site	GPS coordinates		Site intervals	Sampling site distance intervals (km)
	North (°)	West (°)		
S_1_	7.67751	−1.87233	S_1_	0
S_2_	7.61532	−1.91023	S_1_-S_2_	7.283
S_3_	7.55001	−1.95143	S_2_-S_3_	7.727
S_4_	7.45963	−1.94125	S_3_-S_4_	9.096
S_5_	7.27958	−2.26844	S_4_-S_5_	37.35
S_6_	7.05365	−2.31737	S_5_-S_6_	23.12
S_7_	6.96822	−2.32827	S_6_-S_7_	8.612
S_8_	6.80694	−2.42809	S_7_-S_8_	18.97
S_9_	6.61289	−2.39906	S_8_-S_9_	19.62

Source: Nyantakyi et al. [29].

**Table 2:** Precision and accuracy.

Pesticides	0.01 (mg/L)		0.05 (mg/L)			0.01 mg/kg		0.05 mg/kg		
	Mean recovery	RSD (%)	Mean recovery	RSD (%)	Precision intermediate (%)	Mean recovery	RSD (%)	Mean recovery	RSD (%)	Precision intermediate (%)
Parathion	98.1	9.9	101	8.8	11	101.1	8.6	102.1	10.1	10.8
Methamidophos	97.8	10.1	104	8.5	10.5	102.8	8.9	101.8	10	10.2
Diazinon	101.0	8.9	99.2	9.9	10.2	98.9	9.4	99.2	9.9	10.1
Fenitrothion	103.1	7.6	98.0	10	10.1	103	10	101	8.3	9.9
Malathion	98.3	10.3	99.5	8.9	10.4	98.7	8.6	99.3	9.4	10.0
Chlorpyrifos	99.0	9.0	101	10	9.8	99.3	9.3	98.4	10.2	7.8
Profenofos	98.1	9.5	99.7	8.9	10.1	101	8.9	102	9.9	9.21
Pirimiphosmethyl	103.5	8.2	102	9.9	10	99.7	9.9	100.5	9.8	10.2
Allethrin	99.1	8.8	99.6	8.8	10.1	102.1	10.4	103.1	8.5	9.1
Permethrin	98.7	8.3	99.9	9.1	9.9	98.4	10.2	99.7	9.9	8.5
Deltamethrin	99.1	9.2	101	10	10.1	101.9	9.9	101	9.3	10.3
Cyfluthrin	101.5	8.9	103	8.7	10.2	99.5	10.1	103.5	9.9	10
Fenvalerate	104	9.7	103	6.8	8.8	104	10	101	10.1	9.8
*α*-HCH	99.5	9.4	101	8.9	10	99.2	9.4	103.5	10.1	9.4
*β*-HCH	101	9.9	99.9	9.0	9.5	102	9.9	100.5	8.5	10.3
*δ*-HCH	102	10.1	103	10	10.2	101	10	101	8.9	10.1
*γ*-HCH	98.9	10.0	101	10.3	10.4	98.3	9.8	99.9	9.9	10.2
Heptachlor	98.7	9.9	99.7	8.7	8.9	98.1	8.7	99.7	9.7	9.9
Aldrin	102	10.1	101	7.9	10.4	101	9.9	103	9.9	9.4
chlordane	101	9.7	99.8	9.9	10.3	103	9.7	102	10.2	9.1
*α*-Endosulfan	103.2	9.9	102	8.5	10.4	99.7	8/6	98.2	8.4	8/5
*β*-Endosulfan	98.8	9.6	99.9	10	10.3	101	10	98.8	9.9	8.8
Dieldrin	99.6	10	101	10	10.3	99.8	10.2	98.6	8.7	9.3
Endrin	101.1	10.1	102	9.8	10.4	104	9.9	102.1	10	9.2
p,p-DDT	104	9.8	103	9.4	9.8	102	10	101	10.2	8.6
p,p-DDE	103.1	10.2	102	10	10.3	102	9.8	101.4	8.5	8.6

**Table 3:** Seasonal variations in OP pesticide residues in water and sediment samples.

OPs in water samples				OPs in sediment samples			
Pesticides	Group means ± SD (*μ*g/L)				Group means ± SD (mg/kg)			
	Dry season	Rainy season	*t* value	*p* value	Dry season	Rainy season	*t* value	*p* value
Parathion	0.027 ± 0.02	0.268 ± 0.01	−2.34	0.031^*∗*^	0.013 ± 0.04	0.035 ± 0.03	−2.34	0.028^*∗*^
Methamidophos	0.238 ± 0.04	0.241 ± 0.03	−0.02	0.985	0.009 ± 0.01	0.039 ± 0.01	−3.20	0.004^*∗*^
Diazinon	0.024 ± 0.01	0.063 ± 0.05	−1.57	0.127	0.023 ± 0.01	0.023 ± 0.02	0.034	0.973
Fenitrothion	0.021 ± 0.02	0.134 ± 0.04	−1.49	0.154	0.027 ± 0.05	0.052 ± 0.04	−1.26	0.220
Malathion	0.131 ± 0.05	0.303 ± 0.01	−1.07	0.294	0.027 ± 0.02	0.036 ± 0.01	−0.436	0.666
Chlorpyrifos	0.148 ± 0.03	0.383 ± 0.01	−1.32	0.200	0.017 ± 0.00	0.021 ± 0.03	−0.517	0.608
Profenofos	0.074 ± 0.04	0.303 ± 0.07	−1.83	0.079	0.026 ± 0.01	0.021 ± 0.02	0.423	0.673
Pirimiphosmethyl	0.188 ± 0.14	0.309 ± 0.01	−0.62	0.539	0.013 ± 0.04	0.035 ± 0.03	−2.34	0.028^*∗*^

^*∗*^means the seasonal difference is statistically significant (*p* < 0.05)

**Table 4:** Seasonal variations in synthetic pyrethroid pesticide (SPP) residues in water and sediment samples.

SPP in water					SPP in sediment			
Pesticides	Group means ± SD (*μ*g/L)				Group means ± SD (mg/kg)			
	Dry season	Rainy season	*t* value	*p* value	Dry season	Rainy season	*t* value	*p* value
Allethrin	0.012 ± 0.01	0.003 ± 0.03	−3.38	0.002^*∗*^	0.009 ± 0.01	0.012 ± 0.02	−0.612	0.545
Permethrin	0.001 ± 0.05	0.019 ± 0.02	−4.50	0.004^*∗*^	0.008 ± 0.02	0.007 ± 0.01	0.245	0.808
Deltamethrin	0.002 ± 0.02	0.012 ± 0.02	−2.84	0.008^*∗*^	0.004 ± 0.01	0.004 ± 0.01	0.000	1.00
Cyfluthrin	0.002 ± 0.01	0.008 ± 0.01	−2.55	0.016^*∗*^	0.001 ± 0.01	0.001 ± 0.03	−0.589	0.560
Fenvalerate	0.001 ± 0.03	0.007 ± 0.01	−1.91	0.065	0.007 ± 0.01	0.004 ± 0.01	−0.570	0.572

^*∗*^ means difference is significant at *p* < 0.05

**Table 5:** Seasonal variations in OCP residues in water and sediment samples.

OCPs in water					OCPs in sediment			
Pesticides	Group means ± SD (*μ*g/L)				Group means ± SD (mg/kg)			
	Dry season	Rainy season	*t* value	*p* value	Dry season	Rainy season	*t* value	*p* value
*α*-HCH	<0.01	<0.01	N/A	N/A	<0.01	<0.01	N/A	N/A
*β*-HCH	<0.01	<0.01	N/A	N/A	<0.01	<0.01	N/A	N/A
*δ*-HCH	<0.01	0.059 ± 0.24	−1.062	0.296	<0.01	0.004 ± 0.12	N/A	−1.00
*γ*-HCH	<0.01	0.002 ± 0.01	−1.000	0.324	<0.01	0.003 ± 0.01	0.037 ± 0.13	−1.10
Heptachlor	<0.01	<0.01	N/A	N/A	<0.01	<0.01	N/A	N/A
Aldrin	<0.01	<0.01	N/A	N/A	<0.01	0.001 ± 0.01	N/A	−1.00
Chlordane	<0.01	<0.01	N/A	N/A	<0.01	<0.01	N/A	N/A
*α*-Endosulfan	<0.01	<0.01	N/A	N/A	<0.01	<0.01	N/A	N/A
*β*-Endosulfan	<0.01	<0.01	N/A	N/A	<0.01	<0.01	N/A	N/A
Dieldrin	<0.01	<0.01	N/A	N/A	<0.01	<0.01	N/A	N/A
Endrin	<0.01	<0.01	N/A	N/A	<0.01	<0.01	N/A	N/A
p,p-DDT	<0.01	<0.01	N/A	N/A	<0.01	<0.01	N/A	N/A
p,p-DDE	<0.01	<0.01	N/A	N/A	<0.01	<0.01	N/A	N/A

N/A means not applicable; <0.01 means lower than the limit of detection

**Table 6:** Eigen values, percentage variability, and cumulative OP residues association

	F1	F2	F3	F4	F5	F6	F7	F8	F9
Eigenvalue	5.455	1.420	0.711	0.491	0.280	0.209	0.173	0.134	0.049
Variability (%)	60.61	16.66	7.895	5.451	3.109	2.322	1.922	1.486	0.543
Cumulative (%)	60.61	77.27	85.17	90.62	93.73	96.05	97.97	99.46	100.00

## Data Availability

Data of this research can be made available upon request.
